RETRACTED

# Correlation and Prognostic Action of SAA, Hcy, and BNP Levels with the Condition of Patients with Spontaneous Intracerebral Hemorrhage

**DOI:** 10.1155/2022/1126611

**Published:** 2022-06-27

**Authors:** Weiwei Xu, Jing Wang, Hong Yang

**Affiliations:** ^1^The Nanhua Affiliated Hospital, Department of Neurosurgery, Hengyang Medical School, Universitity of South China, Hengyang, Hunan 421001, China; ^2^The Nanhua Affiliated Hospital, Department of Spinal Surgery, Hengyang Medical School, Universitity of South China, Hengyang, Hunan 421001, China; ^3^The Affiliated Nanhua Hospital, Office of Educational Administration, Health School of Neuclear Industry, Hengyang, Hunan 421001, China

## Abstract

**Objective:**

To explore the correlation of serum amyloid A (SAA), homocysteine (Hcy), and plasma B-type brain natriuretic peptide (BNP) levels in patients with spontaneous intracerebral hemorrhage (SICH) and their predictive value for the status and prognosis of SICH patients.

**Methods:**

82 SICH patients admitted to our hospital from March 2017 to March 2020 were selected. According to the Glasgow coma scale (GCS) score, the patients were divided into GCS > 8 group (*n* = 44) and the GCS ≤ 8 group (*n* = 38). Based on the bleeding volume, the patients were divided into the massive bleeding group (>30 ml) (*n* = 21), the moderate bleeding group (10∼30 ml) (*n* = 28), and the small bleeding group (<10 ml) (*n* = 33). Based on the prognostic status of patients after 28 days of admission, they were divided into the survival group (*n* = 64) and the death group (*n* = 18). Serum SAA, Hcy, and plasma BNP levels of patients in different groups were compared, and the correlation between serum SAA, Hcy and plasma BNP levels with GCS score, cerebral hemorrhage, and the prognostic value of patients was analyzed.

**Results:**

Serum SAA, Hcy, and plasma BNP levels in patients with GCS ≤ 8 groups were higher than those in GCS > 8 groups (*P* < 0.05). Serum SAA, Hcy, and plasma BNP levels of patients in the massive bleeding group were higher than those in the moderate and small bleeding groups. Besides, the level of serum SAA, Hcy, and plasma BNP in the moderate bleeding group was higher than that in the small bleeding group (*P* < 0.05). Serum SAA, Hcy and plasma BNP levels of patients were negatively correlated with GCS scores but positively correlated with bleeding volume (*P* < 0.05). The levels of serum SAA, Hcy and plasma BNP in dead patients were higher than those in the survival patients (*P* < 0.05). The combined prediction of serum SAA, Hcy, and plasma BNP for the prognosis of SICH patients was 0.910 (95% CI: 0.984∼0.837), which was higher than the serum SAA, Hcy, and plasma BNP alone predicted AUC 0.679 (95% CI: 0.564∼0.795), 0.720 (95% CI: 0.603∼0.836), and 0.726 (95% CI: 0.616∼0.849).

RETRACTED

**Conclusion:**

The levels of serum SAA, Hcy, and plasma BNP have a correlation with the severity and prognosis of patients with SICH, which is a feasible index for judging the prognosis of SICH. The levels of serum SAA, Hcy, and plasma BNP are conducive to timely judgment of the progression and prognosis of SICH patients.

## 1. Introduction

Spontaneous intracerebral hemorrhage (SICH) is a nontraumatic cerebral parenchymal hemorrhage with complex pathogenesis and severe progression. SICH is characterized by high morbidity, mortality, and disability rates, which affect the quality of life of patients and brings a heavy burden to their families and society [1]. Amyloid A (SAA) is a highly sensitive protein produced by macrophages and fibroblasts activated in the liver in the acute phase of the disease [2]. Studies have shown that SAA rises sharply in the early phase of inflammatory response, which is considered to be involved in the process of arteriosclerosis in cerebrovascular diseases and is critical for the prognosis of cerebral infarction and other diseases [3]. Homocysteine (Hcy), a sulfur-containing amino acid mainly produced by red blood cells, is involved in the secondary damage of acute cerebral hemorrhage and is a key independent risk factor for cardiovascular and cerebrovascular diseases [4]. B-type brain natriuretic peptide (BNP) belongs to the neurohormones and is widely present in cardiomyocytes and brain tissue. The concentration of BNP fluctuates significantly in subarachnoid hemorrhage and acute traumatic brain injury, which is closely related to disease progression [5]. In this study, by measuring the levels of serum SAA, Hcy, and plasma BNP in patients with SICH, we explored the correlation relationship between SAA, Hcy, and BNP with the condition of SICH patients and their predictive effect on the prognosis of patients with SICH.

## 2. Materials and Methods

### 2.1. General Information

A total of 82 SICH patients admitted to our hospital from March 2017 to March 2020 were selected, including 52 males and 30 females, with an average age of 63.28 ± 8.16 years. Head CT examination showed the location of hematoma in patients: 23 cases were located in the left basal ganglia, 39 cases were located in the right basal ganglia, and 20 cases were located in the lobe of the brain. The average blood loss was 19.52 ± 10.21 ml. Inclusion criteria: in line with the “Guidelines for Diagnosis and Treatment of Cerebral Hemorrhage in China (2014)” [6]; The patient was admitted to the hospital within 12 hours of onset, and was confirmed to be SICH by immediate head CT examination; only medical treatment was performed; clinical data and follow-up data were complete. Exclusion criteria: bleeding into the ventricle; history of previous stroke or traumatic brain injury; complicated with dysfunction of vital organs such as the heart, lung, liver, and kidney; died within 24 hours of admission or received surgical treatment due to the changes in condition during the observation period. The severity of the patient's condition was evaluated according to the Glasgow coma scale (GCS) score and the amount of bleeding. According to the GCS score, 44 cases were grouped with a GCS >8 and 38 cases were grouped with a GCS ≤8. According to the amount of bleeding, they were divided into massive bleeding group (>30 ml), 21 cases; moderate bleeding group (10–30 ml), 28 cases; and small bleeding group (<10 ml), 33 cases. This study was approved by the hospital ethics committee, and all patients and their families voluntarily signed informed consent. Also, the clinical baseline data of 82 patients was statistically insignificant.

RETRACTED

### 2.2. Research Methods

General information such as gender, age, underlying disease, and past history was recorded for all patients upon admission. Immediately after admission, venous blood is drawn from the patient for a routine biochemical examination and GCS scoring. The amount of cerebral hemorrhage is estimated according to the Tada formula for the CT membrane of the patient's head at the time of admission; that is, the amount of bleeding (ml) = the length (cm) of the *π* × the width (cm) × the width (cm) × height (cm)/6. All patients underwent routine medical diagnosis and treatment and were given dehydration to reduce intracranial pressure, control blood pressure, regulate blood sugar, and prevent complications. After 28 days of admission, patients were divided into survival group and death group according to the prognosis of patients.

### 2.3. Observation Indicators

Then, 5 ml of venous blood was drawn from all patients immediately after admission, and serum SAA and Hcy levels were detected by immunoturbidimetry and enzyme-linked immunosorbent assay (ELISA), respectively. Plasma BNP levels were detected by ELISA. All reagents were purchased from Shanghai Yinggong Biotechnology Co., Ltd., and the operations were carried out in strict accordance with the kit instructions. The serum SAA, Hcy, and plasma BNP levels of patients in different groups were compared. The correlations of serum SAA, Hcy, and plasma BNP levels with GCS score and intracerebral hemorrhage and their predictive effects on the prognosis of spontaneous intracerebral hemorrhage were analyzed.

RETRACTED

### 2.4. Statistical Methods

The SPSS 22.0 software was used to process experimental data. Measurement data are expressed as mean ± standard deviation ($\bar{X}\pm S$). Enumeration data are expressed as (%). Pairwise comparisons of measurement data between groups were analyzed by the *t*-test. The multigroup comparison of intergroup metrological data is a one-way ANOVA. Enumeration data were analyzed by the *χ*^2^ test. The test level was *α* = 0.05, and *P* < 0.05 or *P* < 0.01 was considered statistically significant.

## 3. Results

### 3.1. Comparison of Serum SAA, Hcy, and Plasma BNP Levels in Patients with Different GCS Scores

The levels of serum SAA, Hcy, and plasma BNP in the GCS ≤8 group were higher than those in the GCS >8 group, and the differences were statistically significant (*P* < 0.05), as shown in Table 1.

### 3.2. Comparison of Serum SAA, Hcy, and Plasma BNP Levels in Patients with Different Bleeding Volumes

The levels of serum SAA, Hcy, and plasma BNP in the massive hemorrhage group were higher than those in the moderate hemorrhage group and the minor hemorrhage group, and the moderate hemorrhage group was higher than the minor hemorrhage group, and the differences were statistically significant (*P* < 0.05), as shown in Table 2.

### 3.3. Correlation of Serum SAA, Hcy, and Plasma BNP Levels with GCS Score and Bleeding Volume

Serum SAA, Hcy, and plasma BNP levels were negatively correlated with the GCS score (*P* < 0.05) and positively correlated with the bleeding volume (*P* < 0.05), as shown in Table 3.

### 3.4. Comparison of Serum SAA, Hcy, and Plasma BNP Levels between Survival Group and Death Group

After 28 days of admission, 64 patients survived and 18 died. The levels of serum SAA, Hcy, and plasma BNP in the death group were higher than those in the survival group, and the differences were statistically significant (*P* < 0.001), as shown in Table 4.

### 3.5. The Predictive Effect of Serum SAA, Hcy, and Plasma BNP Levels on the Prognosis of Patients with SICH

The combined AUC of serum SAA, Hcy, and plasma BNP in predicting the prognosis of patients with SICH was 0.910 (95% CI: 0.984–0.837), which was higher than the AUC of 0.679 (95% CI: 0.564–0.795) predicted by serum SAA, Hcy, and plasma BNP alone, 0.720 (95% CI: 0.603∼0.836), and 0.726 (95% CI: 0.616∼0.849). The combined sensitivity of serum SAA, Hcy, and plasma BNP in predicting the prognosis of patients with SICH was 92.7%, which was higher than the sensitivities of serum SAA, Hcy, and plasma BNP alone, 81.4%, 86.2%, and 87.9%. The specificity of serum SAA, Hcy, and plasma BNP combined to predict the prognosis of patients with SICH was 87.8%, which was higher than the serum SAA, Hcy, and plasma BNP alone (52.7%, 52.9%, and 65.7%), as shown in Table 5 and Figure 1.

RETRACTED

## 4. Discussion

SICH is a nontraumatic sudden intraparenchymal hemorrhage caused by single or multiple factors, accounting for 10% to 15% of strokes, which is a common acute cerebrovascular disease [7]. The pathological injuries and physiological processes stimulated by the pathogenesis of SICH are complex and changeable, closely related to the response of inflammatory mediators and vasoactive substances [8]. Due to the special location of the disease in patients with SICH, the disease is dangerous, changes rapidly, and the prognosis is poor. Early and timely judgment of the progress of the patients is critical for the treatment [9].

SAA is an acute response protein. The level of SAA changes rapidly in the process of the inflammatory response, which is closely related to the secondary injury of brain tissue after cerebral hemorrhage [10]. Hcy is a vital risk factor for the onset of cardiovascular and cerebrovascular diseases. High Hcy affects the body's coagulation system, disrupts its balance, and further aggravates the symptoms of cerebral hemorrhage [11]. BNP is a cardiac hormone synthesized primarily by cardiomyocytes. Under normal physiological conditions, bnp synthesis and secretion are low, which is an important indicator for the detection of heart failure and coronary artery lesions. The synthesis and secretion of BNP are low under normal physiological conditions. BNP has an effect on diuretic, sodium excretion, vasodilation, and antagonistic renin-angiotensin-aldosterone (RAS) system in the neuroendocrine changes of heart failure [12]. Recent studies have shown that the expression of plasma BNP in patients with traumatic brain injury, etc. is significantly higher than that in healthy people, and the concentration of BNP is positively correlated with the amount of cerebral hemorrhage and the degree of cerebral edema, and also has a correlation with the degree of neurological deficit, suggesting that BNP is useful for the diagnosis and treatment of cerebrovascular diseases [13, 14]. The results of this study showed that levels of serum SAA, Hcy and plasma BNP in the GCS ≤8 groups were higher than those in the GCS >8 groups, and the serum SAA, Hcy, and plasma BNP levels in the massive bleeding group were higher than those in the moderate bleeding group and the minor bleeding group, and the moderate bleeding group was higher than the small bleeding group. It is suggested that the lower GCS score and greater bleeding volume in SICH patients indicate higher serum SAA, Hcy, and plasma BNP levels. Therefore, SAA, Hcy, and BNP are all involved in the pathogenesis of SICH patients, which have possible evaluating capacities for the severity of SICH patients [15].

RETRACTED

Some studies have shown that SAA is involved in the whole process of arteriosclerosis and is closely related to the prognosis and classification of cerebrovascular diseases such as cerebral infarction [16]. Elevated HCY levels in patients with SICH promote oxidative stress in vivo, irritate the vascular wall, which in turn damages the vascular endothelium and accelerates the formation of plaque on the vascular wall and secondary injury in patients with cerebral hemorrhage [17]. During the stressful process of SICH patients, ischemia and hypoxia, hematoma compression, etc. can lead to an increase in BNP secretion [18]. The results of this study showed that serum SAA, Hcy, and plasma BNP levels were negatively correlated with GCS score and positively correlated with bleeding volume, which suggests that serum SAA, Hcy, and plasma BNP levels are significantly correlated with the severity of the patients.

In this study, 82 patients were admitted to the hospital. Twenty-eight days later, 64 patients survived and 18 died. The levels of serum SAA, Hcy, and plasma BNP in the death group were higher than those in the survival group. After the occurrence of SICH, the expression of various inflammatory factors is up-regulated, which aggravates inflammation and induces the death of nerve cells. High levels of SAA have a negative impact on the vascular endothelial function of patients. Meanwhile, Hcy causes damage to vascular endothelial cells. It increases significantly with an increase in the degree of neurological deficits [19, 20]. This study also showed that the combined AUC of serum SAA, Hcy, and plasma BNP in predicting the prognosis of patients with SICH was higher than the independent prediction, and the sensitivity and specificity of the combined prediction of serum SAA, Hcy, and plasma BNP were also higher than those of a single prediction, which suggests serum SAA, Hcy, and plasma BNP levels may be used as feasible indicators for judging the prognosis of SICH and help physicians make corresponding predictions on the prognosis of patients with SICH in the early phase of the disease.

In conclusion, serum SAA, Hcy, and plasma BNP levels have a certain correlation with the severity and prognosis of patients with SICH, and higher serum levels of SAA, Hcy, and plasma BNP indicate the severity of SICH, which are feasible indicators for judging the prognosis of SICH and are conducive to early and timely judgment of the progression and prognosis of SICH patients.

## Figures and Tables

**Figure 1:** ROC curve of serum SAA, Hcy, and plasma BNP levels predicting the prognosis of patients with SICH.

RETRACTED

**Table 1:** Comparison of serum SAA, Hcy, and plasma BNP levels in patients with different GCS scores (*n*, $\bar{X}\pm S$).

Group	Number of cases	SAA (mg/L)	Hcy (*μ*mol/L)	BNP (pg/ml)
GCS > 8 group	44	23.46 ± 5.72	16.41 ± 3.84	86.92 ± 27.61
GCS ≤ 8 group	38	37.84 ± 7.65	26.95 ± 4.92	117.29 ± 31.05
*t* value		9.717	10.884	4.688
*P* value		0.000	0.000	0.000

**Table 2:** Comparison of serum SAA, Hcy, and plasma BNP levels in patients with different bleeding volumes (*n*, $\bar{X}\pm S$).

Group	Number of cases	SAA (mg/L)	Hcy (*μ*mol/L)	BNP (pg/ml)
Minor hemorrhage group	33	22.43 ± 5.07	15.92 ± 4.52	68.37 ± 20.46
Moderate hemorrhage group	28	31.37 ± 6.49^a^	20.64 ± 5.81^a^	92.83 ± 25.17^a^
Massive hemorrhage group	21	40.55 ± 9.13^ab^	27.95 ± 6.37^ab^	163.15 ± 31.54^ab^
*F* value		6.159	5.169	3.428
*P* value		0.000	0.000	0.004

Note: compared with the minor bleeding group, ^a^*P* < 0.05; compared with the moderate bleeding group, ^b^*P* < 0.05.

**Table 3:** Correlation of serum SAA, Hcy, and plasma BNP levels with GCS score and bleeding volume.

Indicator	GCS score		Bleeding volume	
	*r* value	*P* value	*r* value	*P* value
SAA	−0.518	0.018	0.541	0.016
Hcy	−0.553	0.014	0.605	0.011
BNP	−0.665	0.007	0.731	0.003

**Table 4:** Comparison of serum SAA, Hcy, and plasma BNP levels between the survival group and the death group (*n*, $\bar{X}\pm S$).

Group	Number of cases	SAA (mg/L)	Hcy (*μ*mol/L)	BNP (pg/ml)
Survival group	64	26.74 ± 5.18	19.26 ± 4.82	80.35 ± 23.59
Death group	18	42.16 ± 7.32	28.53 ± 6.07	174.39 ± 32.76
*t* value		10.136	6.798	13.655
*P* value		0.000	0.000	0.000

**Table 5:** Predictive effects of serum SAA, Hcy, and plasma BNP levels on the prognosis of patients with SICH (*n*, %).

Indicator	AUC	Asymptotic 95% confidence interval		Best cutoff	Sensitivity (%)	Specificity (%)
		Upper limits	Lower limits			
SAA	0.679	0.564	0.795	0.341	81.4	52.7
Hcy	0.720	0.603	0.836	0.391	86.2	52.9
BNP	0.726	0.616	0.849	0.536	87.9	65.7
Joint forecast	0.910	0.837	0.984	0.805	92.7	87.8

## Data Availability

The data can be obtained from the author upon reasonable request.
